# Application of the Flipped Classroom Mode under Few-Shot Learning in the Teaching of Health Physical Education in Colleges and Universities

**DOI:** 10.1155/2022/1465613

**Published:** 2022-03-11

**Authors:** Huimin Wang, Min Chen

**Affiliations:** ^1^Southwest Minzu University, Chengdu, Sichuan 610041, China; ^2^School of Physical Education, Yulin Normal University, Yulin, Guangxi 537000, China

## Abstract

The flipped classroom is a revolutionary teaching method that reverses the traditional roles of teachers and students, as well as the traditional classroom and after-school schedules. The flipped classroom is currently the most popular English teaching reform, so the design and development must meet the practical needs of college physical education teaching. Subverting the classroom is a highly effective service for college physical education that promotes college physical education quality improvement. The research topic of this study is the application of the flipped classroom teaching model based on few-shot learning in public physical education in ordinary colleges and universities. It analyzes the conceptual advantages of the flipped classroom teaching model based on few-shot learning, combining its benefits with the current common college environment. There are issues in physical education, and a teaching model suitable for public physical education in ordinary colleges and universities is gradually being developed in order to improve students' enthusiasm for independent learning and classroom teaching quality. The flipped classroom teaching model has given rise to new ideas for the construction of a physical education model: first, students' physical learning is no longer limited to the physical education classroom, thanks to the use of network technology to change the learning environment. Teaching resources have been expanded to include many online sports resources, so students' physical learning is no longer limited to the physical education classroom. Students can learn anytime and anywhere, which allows them to continue their education throughout their lives; second, flipped classrooms increase teacher-student interaction and play an important role in re-establishing a harmonious teacher-student teaching relationship: third, online courses help students develop their skills. Autonomous learning's ability to shape students' personalized learning is better suited to the development of students' core literacy.

## 1. Introduction

The purpose, principles, and production process of the few-shot learning design for the general physical education major of college physical education are discussed in this article, which first outlines the general few-shot learning design and development. A typical case is taught in few-shot learning, a general physical education course [1]. The fifth section aims to develop the few-shot learning method, which is currently being used in general physical education teaching at colleges and universities, in conjunction with the flipped classroom teaching mode, in order to carry out actual teaching, strictly control the experiment process, and verify the few-shot learning teaching method. It is more beneficial to assist students in learning about sports technology [2].

Teachers and students use various methods in the teaching process to achieve common teaching goals and complete common teaching tasks, which is referred to as a teaching method. The teaching method chosen has a significant impact on the teaching effect, and different teaching methods have different teaching effects. The current physical education teaching method uses a class teaching system, which makes it difficult to respect student differences and even more difficult to provide personalized instruction [3]. The flipped classroom, on the other hand, is a new type of personalized teaching mode based on few-shot learning in the context of information technology. Students can learn anytime and anywhere using the teaching videos created by teachers, and they can track their progress based on their own understanding ability. Students can interact with one another if they have any doubts or incomprehension while self-studying [4]. Above all, teachers can gain a better understanding of each student's learning situation by receiving feedback from students prior to class. At the same time, teachers can group the students of different learning levels in class or group the students according to their mastery of a specific knowledge point and conduct hierarchical teaching according to the actual situation of each group in a targeted manner, taking into account each of them [5].

This article combines my own experience with few-shot learning, identifies flaws and areas that need to be addressed, and then presents my own insights and prospects for future research into few-shot learning. The traditional teaching method emphasizes the importance of continued training in order to improve technology quality. Excessive learning repetition will inevitably bore students and cause them to lose interest in learning. Few-shot learning, which became popular in the 1990s, helped to solve some of these issues [6]. Few-shot learning is being used in college physical education classes to reflect a more free and flexible teaching method, and the content of few-shot learning is being streamlined [7]. Physical education is a skill-based collective project, so it avoids students' resistance to a large amount of teaching content during the learning process, which reduces the classroom's teaching effect, reduces students' learning efficiency, and prevents students from mastering technical movements. A sense of learned helplessness is produced by weakness [8]. The use of the flipped classroom teaching model has improved the status and performance of physical education, facilitated the continued acquisition of physical skills at the university level, and improved the overall development of quality education. The flipped classroom teaching model promotes the advancement of sports reform, the achievement of student-centered physical education goals, the fulfillment of personal needs, and the development of students' interest in sports learning and practice. This study establishes a new practical physical education teaching model, changes the teaching model and organizational form simultaneously, and increases students' enthusiasm for learning and practice.

## 2. Related Work

In recent years, the research on the flipped classroom teaching model is relatively early, and various theoretical methods are relatively mature. Two high school teachers (Jonathan Berman and Aaron sans) from the United States were unable to use screen recording software to record courseware or lecture audio and upload these materials to the Internet, which made the absent students unable to enjoy the relevant course content. The essence of the flipped classroom is to “reverse” or “flip” the traditional teaching form, that is, to transform the traditional “teaching first and then learning” into “first learning and then teaching.” It is subverting the traditional classroom form and forming new teachers and students. Relationship, this is not only a flip of the teaching form but more importantly, the change of teaching philosophy [9]. At the same time, flipping is just a means. Its real purpose is to leave more time in the classroom for teachers and students to fully communicate and interact, stimulate each other's intellectual potential, and free the teacher from the heavy work of repeated teaching. The time guides students to construct the correct knowledge framework and improve the efficiency of students' learning [10].

Literature [11] found through a large number of tests that human memory capacity is infinite in a sense, but people have limited access to learning and acquiring knowledge. There are too many things to learn, which is more than that from a psychological point of view. People's cognitive ability, in layman's terms, is that they are too greedy to chew. Few-shot learning focuses on its “micro” characteristics, the content is refined, the important and difficult points are prominent, and it is easy to quickly internalize the learned knowledge for personal use.

Few-shot learning, also known as few-shot learning process, is the abbreviation of microvideo network courses, according to literature [12]. It focuses on specific subject knowledge points using microteaching videos as the primary carrier, such as key points, difficult points, and doubts. Designed and developed a new type of contextualized and support for a variety of learning methods of online course resources, such as test sites or teaching links, such as learning activities, themes, experiments, and tasks. “Few-shot learning” is defined by literature [13] as “an online teaching video document aimed at explaining a certain point of knowledge, using short and succinct online videos as the form of expression, with the purpose of learning or teaching applications.” Reference [14] considers “few-shot learning” to be beneficial. It is a type of situational and interesting development carefully designed and developed for a specific subject knowledge or teaching link in order to support a variety of learning methods such as flipped learning, blended learning, mobile learning, and fragmented learning, using short and succinct microteaching videos as the main carrier. The package of scientific and visual learning resources “few-shot learning” or “few-shot learning process” means that the time is less than 10 minutes and there is a clear teaching goal and content, according to literature [15]. A brief, small course aimed at explaining a problem. Microlearning is defined as a new type of learning based on microcontent and media that exist in the new media ecosystem, according to the literature [16]. Microlearning, according to the theory, can learn in a reasonable amount of fragmented time, with flexible learning time, no fixed learning location, and a variety of learning forms, including mobile phones, IPAD micromedia application terminals, and systematic learning microcontent to complete knowledge and skill learning tasks.

Literature [17] believes that few-shot learning is a kind of teaching aid resource, which is the basis for implementing flipped classrooms and the carrier of knowledge transfer. It needs a concise but complete teaching design, and an analysis of the learning situation and teaching purpose must be carried out first. Subject development and the actual needs of students choose the appropriate few-shot learning type, and then make a script recording, plus a series of exercises, tests, and other links, to produce short and concise teaching resources, which is a complete teaching system, and vice versa. The flipped classroom is the way to achieve the purpose of few-shot learning and teaching. Only by combining few-shot learning as a teaching resource, the flipped classroom can be effectively realized. Due to the accelerating pace of today's society, people's purpose of acquiring knowledge is stronger, most of them are to meet current needs. The learning time for a few-shot learning is basically between 5 and 15 minutes, and various fragmented ones can be used. Time to study, make full use of time reasonably, and the time requirement is not too high. The 60-second organic chemistry course proposed in the literature [18] was originally designed to allow more ordinary people to understand some basic chemistry knowledge in different situations and hope to apply it to other disciplines. This research has laid a good foundation for the future proposal of “few-shot learning.”

Therefore, it is an urgent need to apply the theoretical results of previous studies to practical teaching in an efficient and reasonable manner, and it is also the greatest significance of this thesis. This article takes the application of few-shot learning in the teaching of general physical education courses of college physical education as the research object. Through the analysis of the disciplinary characteristics and teaching goals of the general physical education courses of physical education in colleges and universities, it uses the form of questionnaires to develop the general physical education The investigation of the current teaching situation of the course, and the measurement of the students' various sports indicators related to this research. Based on this, the design and development of few-shot learning and teaching resources are carried out. A comprehensive analysis of the influence of physical exercise attitude is carried out.

## 3. Few-Shot Learning and Flipped Classroom Related Theories

In the context of deep learning, each class requires at least thousands of training samples to saturate the performance of the CNN on the known classes [19, 20]. In addition, the generalization ability of neural networks is weak. When a novel class comes, it is difficult for the model to learn to recognize novel concepts through a small number of labeled samples. However, all of this is not a problem for humans. We humans have the ability to quickly learn from a small number of (single) samples. Even for a five- or six-year-old child, he has never seen a “panda.” After his father showed him a picture of a panda, the child will recognize the dark circles when he arrives at the zoo. The fat animal is called “panda.”

The following sentence “In Australia, humans have never seen a platypus. Humans will recognize a platypus if you show us a picture of one!” is considered as an illustration Ducks, civet cats, fish, and other animals we've seen in our lives represent prior knowledge of knowledge, while the platypus represents the unknown. This prior knowledge of knowledge is referred to as meta-knowledge, and our brain can quickly access it. A quick comparison of the platypus that has never been seen before and this meta-knowledge (there may be some other mental activities, such as visually extracting the features of objects) [21] leads to the conclusion that this one has the beak of a duck and can swim like a fish. The platypus is a new flat-bodied animal. The example in the preceding paragraph grossly undervalued the human brain. I'm just trying to demonstrate how novel concepts and established knowledge are inextricably linked. Of course, if we are completely unfamiliar with something, we need time to learn.  Figure 1 depicts the general flow of the few-shot learning design.

There is a data set *D*, which we divide into two parts: Dbase and Dnovel, which do not overlap. Dbase is the basic training set that we used to train our model, while Dnovel is the test data. As an example, the 5-way 5-shot is considered. Each time Dnovel is tested, 5 classes (meaning 5-way) are collected. If each of these five classes has 100 samples, we will choose 100 samples at random. Among the 100 samples collected, 5 samples are used as the support set, and the remaining samples are used as the query set [22].

The traditional classroom model is to put the knowledge explanation part in the classroom, mainly to explain the teacher in the classroom, which is a complete teaching model; the flipped classroom model is to use Internet technology to liberate the knowledge of knowledge to the Internet. Students complete the teaching ahead of time through self-learning before class, which greatly reduces the teacher's teaching time in the classroom, allowing students more time to think independently, complete their homework, and communicate with each other in the classroom. The flipped classroom model greatly increases the students' “preparatory time,” and teachers must do their best to achieve the high efficiency of “class time” [23]. The flipped classroom model is shown in Figure 2.

The role of the classroom has changed. In this mode, the teacher has changed from the former classroom teacher to the student's classroom coach. The change in the roles of teachers and students has greatly increased the students' interest in learning, making them more active, profound, interesting in their learning, and more proficient in sports training techniques and improving the quality of learning. In the traditional teaching model, the teacher is the center of the entire class. In the classroom, teachers mainly explain knowledge, while students passively accept knowledge [24]. Due to the lack of interaction and communication, students have lost interest in physical education. However, under the flipped classroom teaching model, the roles of teachers and students have undergone great changes, and students have gradually become the center of the entire class. This is the exchange and discussion of students in the classroom, and the teacher guides and answers questions. In the whole teaching process, teachers only need to control the learning process of students, and when appropriate, divide students into several study groups for communication, discussion, and learning. Students not only learn knowledge but also improve their ability to operate sports techniques.

Few-shot learning is a type of educational resource. It serves as the foundation and knowledge transfer vehicle for flipped classroom implementation. It necessitates a concise but comprehensive teaching strategy. It must first assess the academic situation and teaching purpose in light of the subject's development and the students' current situation. To create short and concise teaching resources, you must first choose the appropriate few-shot type, then record a script, as well as a series of exercises, tests, and other activities, to create a complete teaching system. As a result, the flipped classroom is a one-shot deal. To effectively realize the flipped classroom, the method for achieving the teaching purpose must be combined with few-shot learning, a teaching resource. According to cognitive load theory, the human cognitive structure is made up of short-term and long-term memory. Working memory is another name for short-term memory. It has a very limited capacity. It can only store 5–9 pieces of basic data in most cases. The cognitive load will be exceeded if there is too much learning content. As a result, few-shot learning was born. It is based on small, refined learning content that follows the cognitive load theory and is gradually applied to various teaching methods.

## 4. Design and Practical Application of PE Teaching Model Based on Few-Shot Learning Flipped Classroom Model

The activities of teachers in the preclass stage are mainly the collection of teaching resources and the production of microvideos. Microvideos are mostly the key and difficult points in the teaching content. Therefore, teachers should formulate teaching goals and select teaching content according to the actual situation of students when making. At the same time, it is necessary to consider the individual differences of students, make multiple versions of videos, and explain the teaching content to different levels in a targeted manner. Detailed learning tasks are arranged, a variety of practice methods is provided, and students' problems in the learning process are collected. In the preclass stage, students mainly study independently on the teaching videos provided by the teacher and complete the tasks assigned by the teacher. First, a solution to the problems arising in the study is addressed or discussed and communicated between teachers and students, and between students and students through online platforms. The preclass stage mainly stimulates students' interest in learning and cultivates students' awareness and ability of independent learning, independent thinking, problem-solving ability, and innovative ability. The physical education teaching model design of the flipped classroom model based on few-shot learning is shown in Figure 3.

In the course of the class, the teacher mainly explains and demonstrates the problems that students have before class, organizes students to discuss and practice in groups, and corrects students' wrong actions in time during the tour guide. Students relearn what they have learned in the classroom to achieve knowledge internalization. In the middle of the class, the group discussion exercises mainly cultivate the students' unity and cooperation ability and language organization ability. The skill display link not only cultivates the students' sense of competition but also exercises the students' psychological quality. After class, teachers mainly reflect on the effect of classroom teaching and further improve and optimize the teaching plan. The main purpose is to improve teaching quality and improve student learning efficiency. Students' relearning after class is mainly to consolidate knowledge and further improve their technical level. The after-school period mainly cultivates students' good study habits and develops the consciousness of lifelong sports.

Teaching evaluation is the process of evaluating the process of teaching activities and results using certain standards and methods based on the teaching goals, that is, evaluating the process of teaching activities and results. Its purpose is to make course, teaching, and student training program decisions, with the most important aspect being to evaluate students' academic performance. Traditional teaching evaluation is primarily summative, that is, the assessment of students' learning outcomes at the end of each learning stage. This method focuses on assessing students' mastery of the curriculum, and while the generalization level is high, it may lead students to believe that they do not work hard in normal circumstances. During the exam, the “scallop effect” appears, which is not conducive to boosting students' learning motivation and forming a positive learning outlook.

When teaching evaluation is based on the few-shot teaching method, it uses a teaching evaluation method that is consistent with quality education, focusing on the developmental evaluation of students, and the overall development of student quality is used as the evaluation index. The fundamental principle is that each individual is responsible for his or her own actions. A student's development is based on the student's previous experiences, with a focus on the student's current situation and a greater emphasis on the student's future. The identification of learning levels and the description of student development characteristics are for the future development of students, with a focus on student evaluation in the learning process. Encouragement evaluation is carried out in the classroom, and students' classroom performance is factored into the evaluation of their academic performance. Among them, the timely, quality, and quantity completion of the after-school homework arranged by the teacher is also included in the student's score, that is, after each class, after the smashing skills are strengthened after the class, it is for everyone to communicate and evaluate and give extra points to active students. This evaluation method can not only provide timely feedback through teacher and student comments and help students improve their motor skills, but it can also promote students' subjective initiative and increase their motivation to learn.

## 5. Experimental Process and Design

### 5.1. Academic Analysis

Few-shot learning and instructional design is different from traditional instructional design. At the beginning of the design, it must take into account its short and powerful characteristics and highlight its original intention of explaining the important and difficult points. Compared with traditional teaching methods, few-shot learning with the help of videos, animations, and exquisite diagrams can attract the attention of students, increase their interest in learning, ignite their passion, stimulate their vitality in learning this sport, let them enjoy learning basic knowledge and skills and action methods in a happy atmosphere and learning by playing and playing while learning, constantly stimulate their potential, mobilize students' enthusiasm and subjective initiative in learning, and let them experience the joy of success through the learning of technical movements.

Before the teaching experiment, the subjects were surveyed with relevant questionnaires, and the survey results are shown in Figure 4.

It can be seen that the new teaching method is supported and welcomed by the students. At the same time, in the questionnaire survey, the learners' learning attitudes are analyzed, and when they have poor skills or technical actions that are not well understood in the learning process, which solutions students prefer, the results of the survey are shown in Figure 5:

In the process of students learning in the past teaching methods, 83.33% of the students tend to ask the teacher and 11.67% of the students choose to watch the teaching video. Although these data are relatively small, it can be seen Although the number of samples we collected is relatively small, it can be seen from the results that the flipped classroom teaching model meets the requirements of current students' learning.

## 6. Instructional Design

This article randomly selects students from eight classes of the same grade. The body shape and physical fitness are used as the breakthrough test data to explain the problem, the four classes with no significant differences are chosen as the experimental class, and the other four classes are chosen as the control class. The experiment class adopts the new teaching mode of flipped classroom, and the control class adopts the traditional teaching mode. Finally, the collected data were compared and the relevant data during the experiment was recorded.

Through the analysis of the pretest data of the experimental class and the control class, as shown in Figure 6.

The test data include height, weight, 50 m, and sit-ups (female) items. The data index *t*-test before the test showed that the *P* value was higher than 0.05, indicating that the experimental group and the control group had no significant differences in body shape and physical quality.

The data of students' physical fitness after training can be obtained from Figure 7.

The precheck items of human body shape and athletic ability were retested after the flipped classroom teaching model experiment. The *P* values are both large after *t*-testing, the height and weight test data are statistically obtained. The results revealed that there was no significant difference between the experimental and control groups' test results.

## 7. Significance Analysis of Attitudes toward Physical Training after Experimental Class and Control Class

After one semester of physical education, both classes have basically completed the smash and serve skills. At the same time, the physical exercise attitude of the two classes was investigated. The *t*-test was used to reflect the physical exercise attitude before and after the two semesters. Change, the difference in physical exercise attitude between the two classes, is shown in Tables 1 and 2. The corresponding results can be found in Figures 8–11.

Through analysis, it can be seen that the control class's attitude toward physical activity has slightly changed, whereas the experimental class's attitude toward physical activity has greatly improved, owing to the fact that the new teaching method is relatively new and the teaching method is relatively new. It is one of a kind and better suited to their learning styles. In conclusion, few-shot learning combined with a flipped classroom teaching mode has a greater impact on improving students' physical exercise attitudes than traditional teaching methods, resulting in increased physical activity behavior. This demonstrates that few-shot learning combined with the flipped classroom teaching mode can effectively improve students' basic level and their spiking skills. For middle-level students, both teaching methods have improved and the degree of improvement has increased. Few-shot learning combined with flipped classroom teaching mode is almost as good as traditional teaching methods in terms of improving students' high-level learning.

It was found that the physical fitness of the two classes had improved before and after the experiment. This was an inevitable result of one semester of sports training, and the improvement of the physical fitness of the two classes was roughly the same. This shows that this teaching method and traditional teaching methods are improving students There is no obvious advantage in physical fitness. The reason is that physical education has a lot of content and heavy tasks. In the teaching process, the teacher focuses more on skills and skills teaching and does not carry out special physical fitness exercises.

## 8. Conclusions

Both the school leaders and the teachers themselves must attach importance to the learning of few-shot learning and production technology and vigorously promote the use of few-shot learning and educational resources, but we should also pay attention to the effectiveness of the above methods in practical application. At the same time, the school should regularly invite few-shot learning and production experts to train all teachers, so that teachers can master the technology as soon as possible and complete the teaching tasks with quality and quantity.

When teaching evaluation is based on the few-shot learning and teaching method, it uses a teaching evaluation method that is consistent with quality education, focusing on the developmental evaluation of students and using the overall development of student quality as the evaluation index. The fundamental principle pertains to a student's development. Teachers who are quick to accept can help other teachers form a learning environment of mutual help and mutual assistance based on their own experience and expertise resource and encourage teachers to develop their own style of few-shot learning education based on their own experience and expertise resource. Furthermore, in order to more effectively share teaching resources, schools should create a few-shot learning and education resource information sharing platform as soon as possible to maximize information sharing. The traditional teaching method limits the assessment of students' learning to a review of their theoretical knowledge and skills. The evaluation method is relatively simple, which is detrimental to students' overall development. As a result, the content of future learning evaluations will be more diverse. The performance of students' affection and sense of cooperation should be given more attention. Similarly, evaluation methods should be varied, and a combination of methods can be used to make an objective and fair assessment of students' learning situations. It is based on the student's previous experiences, with a focus on the student's current situation and a greater emphasis on the student's future. The identification of learning levels and the description of student development characteristics are for the future development of students, with a focus on student evaluation in the learning process. Encouragement evaluation is carried out in the classroom, and students' classroom performance is factored into the evaluation of their academic performance. Students who are active will receive extra points for completing after-school homework on time, in a good quality and in a quantity that the teacher has assigned. This evaluation method can not only provide timely feedback through teacher and student comments and help students improve their motor skills, but it can also promote students' subjective initiative and increase their motivation to learn.

The teaching time for this experiment is relatively short for a variety of reasons, and there are some important and difficult points that students do not fully grasp. Simultaneously, the number of samples in the teaching experiment should be increased to make it more convincing. The use of this teaching method is encouraged.

## Figures and Tables

**Figure 1:** Few-shot learning design process.

**Figure 2:** Flipped classroom mode.

**Figure 3:** The design process of physical education model.

**Figure 4:** Attitudes toward physical education.

**Figure 5:** Students' problem-solving methods.

**Figure 6:** The physical condition of the students before the experiment.

**Figure 7:** The physical fitness of students after training.

**Figure 8:** The average value of students' attitudes toward physical exercise before and after the experiment in the experimental class.

**Figure 9:** The standard deviation of students' physical exercise attitude before and after the experiment in the experimental class.

**Figure 10:** Mean values of students' physical exercise attitudes before and after the experiment in the control class.

**Figure 11:** Standard deviation of students' physical exercise attitude before and after the experiment in the control class.

**Table 1:** The analysis of the students' attitudes toward physical exercise before and after the experiment in the experimental class.

	Before the experiment		After the experiment	
	Mean	Standard deviation	Mean	Standard deviation
Action	27.58	4.37	28.78	5.42
Manner	41.89	6.05	45.95	7.39
Cognition	26.42	4.30	28.13	4.76
Habit	32.31	6.25	34.29	7.61
Emotion	31.72	4.81	23.81	5.40
Standard deviation	24.38	4.49	24.97	5.35
Intention	25.03	3.69	26.21	4.31
Subjective goal	20.03	3.32	20.11	3.61

**Table 2:** Analysis of students' attitudes toward physical exercise before and after the experiment in the control class.

	Before the experiment		After the experiment	
	Mean	Standard deviation	Mean	Standard deviation
Action	28.03	5.25	28.06	5.45
Manner	43.64	19.48	43.92	7.76
Cognition	26.02	4.13	26.67	5.21
Habit	33.54	8.61	32.56	7.61
Emotion	34.77	6.54	34.81	6.78
Standard deviation	24.21	3.71	23.84	5.72
Intention	25.31	4.39	24.89	4.67
Subjective goal	21.54	4.05	20.45	4.02

## Data Availability

The dataset used to support the findings of this study is available from the corresponding author upon request.
